The article "Mechanism of Yangxin Tongmai Decoction in the Treatment of Coronary Heart Disease with Blood Stasis Syndrome Based on Network Pharmacology and Molecular Docking" was published in 2022. Journal: Evid Based Complement Alternat Med.

# Mechanism of Yangxin Tongmai Decoction in the Treatment of Coronary Heart Disease with Blood Stasis Syndrome Based on Network Pharmacology and Molecular Docking

**DOI:** 10.1155/2022/4692217

**Published:** 2022-09-30

**Authors:** Mengxue Zhang, Jia Liu, Xiangzhuo Zhang, Shumeng Zhang, Yujie Jiang, Zixuan Yu, Ting Xie, Yuxia Chen, Lingli Chen, Jie Li

**Affiliations:** ^1^Hunan University of Traditional Chinese Medicine, Hunan Changsha 410208, China; ^2^Longhua Hospital, Shanghai University of Traditional Chinese Medicine, Shanghai 200032, China; ^3^Hunan Provincial Key Laboratory of Pathogenic Biology Based on Integrated Chinese and Western Medicine, Hunan University of Chinese Medicine, Hunan Changsha 410208, China

## Abstract

This study aimed to explore the mechanism of Yangxin Tongmai decoction (YXTMD) in the treatment of coronary heart disease (CHD) with blood stasis syndrome (BSS) using network pharmacology and molecular docking, and to verify these results through clinical trials. The active compounds of YXTMD were identified using the Traditional Chinese Medicine Systems Pharmacology database, and the targets of the active compounds were predicted using the SwissTarget Prediction database. The targets of CHD and BSS were predicted using the GeneCards, OMIM, PharmGKB, TTD, and DrugBank databases. The common targets of “herb-disease-phenotype” were obtained using a Venn diagram, then used Cytoscape software 3.8.2 and its plug-in CytoNCA and STRING database to construct the “herb active compounds-common target” and protein–protein interaction networks. R language software and bioconductor plug-in were used for Gene Ontology (GO) and Kyoto Encyclopedia of Genes and Genomes (KEGG) enrichment analyses. AutoDock was used for the molecular docking analysis. Finally, clinical trials were conducted to confirm the results of network pharmacology. Eighty-three active components were obtained, and the core active components were 5,7,4′-trimethoxyflavone, tetramethoxyluteolin, isosinensetin, sinensetin, and 5,7-dihydroxy-2-(3-hydroxy-4-methoxyphenyl)chroman-4-one. A total of 140 common targets were identified, and the core targets were EGFR, VEGFA, AKT1, STAT3, TP53, ERBB2, and PIK3CA. Biological processes identified by the GO analysis primarily involved wound healing, regulation of body fluid levels, and vascular process in circulatory system. The cellular components were primarily located in the membrane raft, membrane microdomain, and plasma membrane raft. The primary molecular functions were activity of transmembrane receptor protein kinase, transmembrane receptor protein tyrosine kinase, and protein tyrosine kinase. KEGG analysis showed that the PI3K-Akt signaling pathway was closely related to the treatment of CHD with BSS by YXTMD. Molecular docking results showed that the core active components had a good binding activity with the core targets. The clinical trial results showed that YXTMD improved the BSS scores and decreased the serum levels of total cholesterol and low-density lipoprotein cholesterol. Moreover, the levels of *PI3k* and *AKt* mRNA were upregulated and the levels of *GSK-3β* mRNA were downregulated. YXTMD has multicomponent, multitarget, and multipathway effects in the treatment of CHD with BSS, and its mechanism of action may involve activation of the PI3K-AKt signaling pathway, downregulation of GSK-3*β*, and mediation of in vivo lipid metabolism-based metabolic processes.

## 1. Introduction

Coronary heart disease (CHD) is caused by coronary artery atherosclerosis or spasms. This condition triggers stenosis or occlusion of the lumen, resulting in myocardial ischemia and hypoxia as well as clinical symptoms such as chest pain and tightness [1]. The World Health Organization (WHO) estimated that the number of people who died of cardiovascular disease worldwide accounted for approximately one-third of all deaths in 2019, among which ischemic heart disease was the most common [2]. The morbidity and mortality rates of CHD are likely to continue to grow due to the aging of the population, thereby seriously threatening human health and becoming a global public health burden [3]. The main clinical treatment for this disease is drug therapy, including lipid-regulating and stabilizing drugs, antiplatelet aggregation and thrombosis drugs, anticoagulant drugs, nitrate drugs, and *β*-receptor blockers [4]. Although these drugs can improve symptoms and delay disease progression, they have a single target of action and drug combinations are often required. Some patients also experience side effects after long-term use, such as liver and kidney function damage, bleeding, and hypotension [5, 6]. Therefore, other therapeutic drugs still need to be actively explored.

A wide range of Chinese herbal medicines exist with fewer toxic side effects than western medicine [7, 8]. They have the characteristics of being multicomponent, multitarget, and multipathway in the treatment of diseases, which can compensate for the limitations of a single Western medical treatment. In particular, Chinese herbal medicines have unique advantages in preventing and treating CHD [9, 10]. At the same time, it can reduce the side effects of Western medicine [11]. CHD belongs to the traditional Chinese medicine (TCM) category of “chest obstruction, cardiac pain, and genuine heart pain,” and its key pathogenesis is “the obstruction of cardiac vessels (Xin Mai Bu Tong).” The principle of TCM is “discriminatory treatment.” With the increasing number of studies on TCM syndromes, more researchers are exploring new ways to treat diseases from this perspective. Blood stasis syndrome (BSS) is the most common type of CHD [12] and is a research hotspot in the current mode of disease-syndrome combination. Yangxin Tongmai decoction (YXTMD) was developed by a renowned TCM physician, Mr. Bowei Qin, and is an effective prescription for treating cardiovascular diseases [13]. Subsequently, Professor Zhaokai Yuan modified it according to the theory of “nourishing heart Qi (Fu Yang Xin Qi) and re-establishing blood circulation (He Tong Xue Mai).” YXTMD comprises five drugs: renshen (Radix Ginseng), guizhi (Ramulus Cinnamomi), danshen (Radix Salviae Miltiorrhizae), zhishi (Fructus Aurantii Immaturus), and zexie (Rhizoma Alismatis). Preliminary clinical and experimental studies have confirmed that YXTMD prescription can relieve angina pectoris and antimyocardial ischemia, lower blood lipids, inhibit inflammatory response, activate platelet aggregation, promote coronary angiogenesis, and increase coronary blood flow [14–16]. Although the therapeutic effect of YXTMD is exact, its main active ingredients and mechanisms of action in the treatment of CHD with BSS have not been fully clarified due to its multitarget action.

Network pharmacology is used to study drugs and their targets and pharmacological activities based on a “drug component–target–disease” interaction network. This network can clarify the mechanism of action of drugs in the treatment of diseases from a holistic perspective and provide new ideas for research on Chinese herbal medicines and their compounds. We therefore aimed to explore the active ingredients, key targets, and specific mechanisms of action of YXTMD in the treatment of CHD with BSS using network pharmacology and molecular docking technology. These results were further verified in clinical trials to provide a theoretical basis for the development and clinical application of the drug. The detailed workflow of the study is shown in Figure 1.

## 2. Materials and Methods

### 2.1. Active Compounds and Targets of YXTMD

The Traditional Chinese Medicine Systems Pharmacology (TCMSP) database [17] (https://tcmspw.com/tcmsp.php) was used to identify the chemical components of YXTMD, including renshen, guizhi, danshen, zhishi, and zexie. Oral-bioavailability (OB) [18] ≥30% and drug-likeness (DL) [19] ≥0.18 were used as parameters to determine the active compounds of YXTMD. The PubChem [20] (https://pubchem.ncbi.nlm.nih.gov/) database was used to collect and collate candidate compounds, and the data were saved in SDF format as 2D or 3D structures. Swisstarget prediction [21] (https://www.swisstargetprediction.ch/) was used to predict the target of the active compounds by setting the species as “Homo sapiens.” Meanwhile, compounds without chemical structures and targets were eliminated, and the UniProt (https://www.uniprot.org/) database was used to standardize potential targets.

### 2.2. Targets of CHD with BSS and Common Targets of “YXTMD-CHD-BBS”

The GeneCards (https://www.genecards.org/), OMIM (https://omim.org/), PharmGkb (https://www.pharmgkb.org/), Therapeutic Target (TTD) (https://db.idrblab.net/ttd/), and DrugBank (https://www.drugbank.ca/) databases were used to collect the targets of the disease and phenotype. We set “coronary heart disease” and “blood stasis syndrome” as the keywords. Related target genes were merged and duplicate values removed to obtain the related targets of CHD with BSS. The common targets of “YXTMD-CHD-BBS” were obtained using VandePeer Labin Bioinformatics Gent (https://bioinformatics.psb.ugent.be/beg), and a Venn diagram was drawn.

### 2.3. Network Construction of “Active Components of YXTMD-Common Targets”

Cytoscape 3.8.2 software was used to construct a network model of “active components of YXTMD-common targets.” The network diagram was analyzed using a network analyzer to obtain the degree ranking of active components.

### 2.4. Protein–Protein Interaction Network

Common targets were imported into the STRING [22] (https://string-db.org/) database, and the research species was set as “*Homo sapiens*.” The minimum confidence score was 0.700 [23] and a network diagram of protein–protein interactions (PPI) was obtained. The protein interaction data were imported into Cytoscape 3.8.2, and the algorithms of betweenness, closeness, degree, eigenvector, and the local average connectivity-based method and network in CytoNCA were used for topological analysis [24]. The core gene was screened

### 2.5. Gene Ontology and Kyoto Encyclopedia of Genes and Genomes Pathway Enrichment Analysis

Gene ontology (GO) and Kyoto Encyclopedia of Genes and Genomes (KEGG) pathway enrichment analyses were performed using R software and the bioconductor plug-in with a screen condition of *P* < 0.05. The top ten items were selected for visualization, and a bar diagram and bubble diagram were drawn.

### 2.6. Molecular Docking

The 2D structures of the active components were downloaded from the PubChem database and saved in mol2 format using ChemBio3D Ultra software. The pdb formats of the 3D structures of the targets were downloaded from the Protein Data Bank (PDB) (https://www.rcsb.org/) based on the core gene target IDs found in the UniProt database. The PyMOL software was used to remove water molecules, and hydrogen atoms were added to the targets. AutoDock software was used to convert the format of active components and target proteins into the pdbqt format. Finally, molecular docking was performed using AutoDock Vina software and the results were visualized using PyMOL software. A binding energy less than “5 kcal/mol” was used to indicate a good binding interaction between the compound and the target [25].

### 2.7. Verification of Clinical Trial

#### 2.7.1. Participants

A total of 26 patients with CHD with BSS admitted to the cardiovascular department of the First Affiliated Hospital of Hunan University of Chinese Medicine between April 2021 and January 2022 were recruited for this study. This study was approved by the Ethics Committee of the First Affiliated Hospital of Hunan University of Chinese Medicine (No. HN-LL-GZR-201820).

1. Diagnostic criteria
2. CHD was diagnosed according to the “Guidelines for the Diagnosis and Treatment of Chronic Stable Angina Pectoris” [26] and “Guidelines for the Diagnosis and Treatment of Unstable Angina Pectoris and Non-ST-elevation Myocardial Infarction” [27] established by the Chinese Medical Association Cardiovascular Branch in 2007. Coronary angiography revealed at least one coronary artery with ≥50% luminal diameter. BSS was diagnosed according to the “Diagnostic Criteria of Coronary Heart Disease with BSS” formulated by the committee of promoting blood circulation and removing blood stasis in 2016 [28].
3. Inclusion criteria
4. Patients who met the above diagnostic criteria for CHD and BSS, had complete clinical data, and voluntarily participated in the study and provided informed consent were included in the study.
5. Exclusion criteria
6. Excluded from the study were patients with severe heart disease (thyroid-related cardiomyopathy, hypertensive heart disease, anemic heart disease, pulmonary heart disease, rheumatic heart disease, etc.); those with malignant tumors, blood system diseases, connective tissue diseases, mental disorders, tuberculosis, and other infectious diseases; those with serious complications of liver and kidney dysfunction; those with poor compliance and incomplete clinical test data; and those who refused to accept the study and provide informed consent.

#### 2.7.2. Main Instruments and Reagents

The following instruments and reagents were used: a fluorescence quantitative PCR instrument; fluorescence PCR plate (Thermo Fisher Scientific, Waltham, MA, USA); desktop freezing centrifuge (Xiangyi, Hunan, China); electrophoresis instrument; horizontal agarose electrophoresis tank (Liuyi, Beijing, China); biological sample homogenizer (Aosheng, Hangzhou, China); enzyme-labeling analyzer (Jiancheng Bioengineering Research Institute, Nanjing, China); ultra-microspectrophotometer (Baoyude Scientific Instrument, Shanghai, China); mRNA reverse-transcription kit (Code No. CW2569; Kangwei Century, Beijing, China); superoxide dismutase (SOD), nitric oxide (NO), and malondialdehyde (MDA) enzyme-linked immunosorbent assay (ELISA) kits (Code No. A001–3, A013-2, and A003-1; Jiancheng Bioengineering Research Institute, Nanjing); tumor necrosis factor-*α* (TNF)-*α* and interleukin-1*β* (IL)-1*β* ELISA kits (Code No. ml077385–2 and ml058059-2;enzyme-linked organisms, Shanghai, China); ethylenediaminetetraacetic acid (EDTA) (Code No. MB2514; Meilun, Dalian, China); Tris (Code No.V900483; Sigma-Aldrich, St. Louis, MO, USA); Trizol (Code No. 15596026; Thermo Fisher Scientific); UltraSYBR (Code No.CW2601; Kangwei Century, Beijing, China); and a blood collection needle and 5 ml blood collection tube (Sanli Medical Technology, China).

#### 2.7.3. Research Methods

1. Trial group
2. Data from 14 eligible patients were collected according to the criteria for diagnosis, inclusion, and exclusion. Patients were divided into two groups according to the random-number table method: the control group (*n* = 7) and the treatment group (*n* = 7). The control group included 5 males and 2 females (average age = 64.14 ± 4.95 years), and the treatment group included 5 males and 2 females (average age = 59.29 ± 5.94 years). No significant differences were observed in the general data between the two groups (*P* > 0.05).
3. Treatment
4. Patients in the control group were administered routine western medicine, including aspirin enteric-coated tablets (100 mg by mouth per day [po qd]), atorvastatin calcium tablets (20 mg po qd), metoprolol succinate sustained-release tablets (23.75 mg po qd), and benazepril hydrochloride tablets (5 mg po qd). Antiangina drugs were discontinued during the treatment period. If angina pectoris broke out, nitroglycerin tablets were administered sublingually as appropriate.
5. Patients in the treatment group were administered YXTMD combined with routine western medicine. The YXTMD comprised Radix Panacis Quinquefolii (6 g), Ramulus Cinnamomi (8 g), Radix Salviae Miltiorrhizae (10 g), Fructus Aurantii Immaturus (10 g), and Rhizoma Alismatis (10 g). All Sanjiu granule types were produced by China Resources Sanjiu Pharmaceutical Co. Ltd. and one dose was administered per day and taken twice.
6. The treatment period for the two groups was 28 days. Patients were evaluated before and after treatment to determine the curative effects of the drugs according to the “Evaluation Criteria of Angina Pectoris and Electrocardiogram in Coronary Heart Disease” [29] and “Efficacy Evaluation Criteria for Coronary Heart Disease Angina Pectoris with Blood Stasis Syndrome” [30].
7. Sample collection
8. Before and after treatment, 12 mL of elbow venous blood was taken from each patient after 8 h of fasting using a red common tube, sodium citrate blood collection tube, and EDTA-K2 anticoagulant blood collection tube. An ice-bag incubator was used to transport the blood samples, of which 4 ml was sent to the biochemical laboratory of the First Affiliated Hospital of Hunan University of Chinese Medicine within 2 h to determine the level of blood lipids. The remaining 8 mL was sent to the Intermediate Diagnosis Laboratory of Hunan University of Chinese Medicine within 2 h; 4 mL was poured into a cryopreservation tube, and the remaining 4 mL was centrifuged. The serum was poured into a cryopreservation tube, and all samples were stored at −80°C.

#### 2.7.4. Index Determination

1. ELISA
2. Blood samples were strictly analyzed according to the manufacturer's instructions. The curve formula was calculated using the standard concentration and absorbance (OD value) of the standard well. The measured OD values were substituted into the corresponding curve formulas to calculate the concentration of MDA, SOD, NO, TNF-*α*, and IL-1*β*.
3. Real-time PCR
4. Total RNA was extracted from the whole blood and reverse transcribed into cDNA. Finally, fluorescence quantitative PCR was performed to determine the expression levels of *PI3k*, *AKt*, *NF-κB*, *eNOS*, and *GSK-3β* mRNA. The steps of the reaction included an initial denaturation at 95°C for 10 min, followed by 40 cycles of denaturation at 95°C for 15 s and annealing at 60°C for 30 s. GAPDH served as an internal control, and gene expression was analyzed by the 2^−ΔΔCt^ method. Primer sequences were designed using Primer 5 and synthesized by Shanghai Bioengineering (Table 1).

#### 2.7.5. Statistical Analysis

SPSS26.0 software was used for statistical analysis. Data are expressed as the mean ± standard deviation ($\bar{x}$ ± *s*). For normally distributed data, the *t*-test was used when the variance was homogeneous and the Wilcoxon test was used when the variance was not homogeneous. Count data are expressed as frequency (constituent ratio,%), and comparisons between two groups were analyzed using the *χ*^2^ test or Fisher's exact test was appropriate. Statistical significance was set at *P* < 0.05.

## 3. Results

### 3.1. Active Components and Related Targets of YXTMD

Using the TCMSP and SwissTarget Prediction databases, the active components of YXTMD were determined, and their related targets were predicted, including for 22 types of renshen, 65 types of danshen, 7 types of guizhi, 22 types of zhishi, and 10 types of zexie. A total of 83 active components and 808 potential related targets were obtained after eliminating compounds without chemical structures or targets and removing repetitive terms.

### 3.2. Common Targets of “YXTMD-CHD-BSS”

Using the GeneCards, OMIM, PharmGkb, TTD, and DrugBank databases, 4003 targets of CHD and 1023 targets of BSS were obtained. Using BioinformaticsGent, 140 common targets were identified at the intersection of “YXTMD-CHD-BSS” (Figure 2).

### 3.3. “YXTMD Active Components-Common Targets” Network

Perl software was used to sort the data, and 83 active components of YXTMD and 140 common targets were obtained. Using Cytoscape 3.8.2 software, the “YXTMD active components-common targets” network was drawn (Figure 3). The network comprises 223 nodes and 1177 edges. The results showed that the top five components were 5,7,4′-trimethylapigenin (degree = 32), tetramethoxyluteolin (degree = 31), isosinensetin (degree = 30), sinensetin (degree = 29), and 5,7-dihydroxy-2-(3-hydroxy-4-methoxyphenyl)chroman-4-one (degree = 28) (Table 2).

### 3.4. “Common Targets” PPI Network

Common targets were imported into the STRING11.5 database to construct the PPI network diagram; isolated nodes were removed (Figure 4(a)). The network contained 140 nodes and 677 edges, with an average clustering coefficient of 0.46. We used the Cytoscape plug-in CytoNCA to screen the key genes (Figure 4(b)) and core genes were integrated using two algorithms (Table 3). According to degree size, the order of the core genes was epidermal growth factor receptor (*EGFR*), vascular endothelial growth factor *(VEGF) A*, *AKT1*, *STAT3*, *TP53*, *ERBB2*, *PIK3CA*, *HSP90AA1*, *mTOR*, *SRC*, *CASP3*, matrix metalloproteinase 9 *(MMP9)*, *IL2*, *NRAS*, *PTPN11*, *TNF*, *PTGS2*, and *FGF2*. These findings indicate that these may be core genes targeted by YXTMD in the treatment of CHD with BSS.

### 3.5. GO Function and KEGG Enrichment Analyses

In total, 2710 were enriched in the GO analysis, including biological processes (BP), cell composition (CC), and molecular function (MF). The top ten items were selected for visualization (Figure 5). BP was primarily concentrated in wound healing, regulation of body fluid levels, vascular progress in the circulatory system, positive regulation of the MAPK cascade, and positive regulation of kinase activity. CC primarily included the membrane raft, membrane microdomain, plasma membrane raft, caveola, apical part of the cell, and apical plasma membrane. MF was primarily concentrated in transmembrane receptor protein kinase activity, transmembrane receptor protein tyrosine kinase activity, protein tyrosine kinase activity, nuclear receptor activity, and ligand-activated transcription factor activity.

A total of 158 signaling pathways were identified by the KEGG enrichment analysis. The top 30 items were selected for visualization (Figure 6), which primarily included the PI3K-Akt signaling pathway, proteoglycans in cancer, Rap1 signaling pathway, MAPK signaling pathway, microRNAs in cancer, and lipids and atherosclerosis. Based on the network pharmacology results and relevant literature [31], we speculated that the PI3K-Akt signaling pathway was closely related to the treatment of CHD with BSS by YXTMD, and therefore visualized the PI3K-Akt signaling pathway (Figure 7).

### 3.6. Molecular Docking

Akt1 plays an important role in vascular remodeling, formation, vasodilation, and wound healing by regulating downstream signaling molecules [32]. In addition, VEGF regulates the proliferation of endothelial cells and promotes angiogenesis through the PI3K-Akt signaling pathway [33]. Accordingly, 5,7,4′-trimethylapigenin, tetramethoxyluteolin, isosinensetin, sinensetin, and 5,7-dihydroxy-2-(3-hydroxy-4-methoxyphenyl)chroman-4-one were selected as the active components for molecular docking with Akt1 and VEGFA (Figure 8).

The results show that the binding energies were less than −5 kcal/mol, indicating that 5,7,4′-trimethylapigenin, tetramethoxyluteolin, isosinensetin, sinensetin, and 5,7-dihydroxy-2-(3-hydroxy-4-methoxyphenyl)chroman-4-one bound strongly to Akt1 and VEGFA (Table 4).

### 3.7. Clinical Trial Results

#### 3.7.1. Efficacy of ECG

Those without abnormal ECG before treatment were excluded from the trial. After treatment, the ECG effective rate of the treatment group was 100%, which was higher than that of control group (50%), but the difference was not significant (*P* > 0.05) (Table 5). The small sample size may have impacted these results.

#### 3.7.2. BSS Scores

No statistically significant differences were found between the two groups before treatment, and the data were comparable. Following treatment, the BSS scores decreased in the treatment group (*P* < 0.05). The BSS score also decreased in the control group, but the difference was not significant (*P* > 0.05). The BSS scores of the treatment group showed a more significant decrease compared with those of the control group after treatment (*P* < 0.05) (Table 6).

#### 3.7.3. Blood Lipids

No statistically significant differences were found between the two groups before treatment, and the data were comparable. The high-density lipoprotein cholesterol (HDL-C) level of the two groups increased after treatment (*P* < 0.05). Total cholesterol (TC), triglyceride (TG), and low-density lipoprotein (LDL) cholesterol (LDL-C) levels were lower in the treatment group, but the difference was not significant (*P* > 0.05); TC and LDL-C levels were higher in the control group (*P* < 0.05). The TC and LDL-C levels of the treatment group showed a greater decrease than those of the after treatment (*P* < 0.05) (Table 7).

#### 3.7.4. Serum Levels of MDA, SOD, NO, IL-1*β*, and TNF-*α*

No statistically significant differences were observed between the two groups before treatment, and the data were comparable. The serum levels of MDA did not significantly change in either group following treatment; the serum levels of SOD and NO were higher in both groups but the difference was not significant (*P* > 0.05). The serum levels of IL-1*β* and TNF-*α* were lower in the treatment group, but the difference was not significant (*P* > 0.05). The serum levels of IL-1*β* were significantly higher in the control group (*P* < 0.05), and although the serum levels of TNF-*α* were also higher, the difference was not significant (*P* > 0.05). Compared with the control group after treatment, no statistical difference was observed in the treatment group (Table 8).

#### 3.7.5. mRNA Levels of *PI3k*, *AKt*, *NF-κB*, *eNOS*, and *GSK-3β*

No statistically significant differences were found between the two groups before treatment, and the data were comparable. The levels of *PI3k*, *AKt*, *NF-κB*, and eNOS mRNA were higher in both groups following treatment (*P* < 0.05). The level of *GSK-3β* mRNA was significantly lower in the treatment group (*P* < 0.05), and although it was lower in the control group, the difference was not significant (*P* > 0.05). Compared with the control group after treatment, the levels of *PI3k* and *AKt* mRNA increased to a greater extent in the treatment group, and the level of GSK-3*β* mRNA decreased significantly (*P* < 0.05) (Table 9). Amplification plots and melting curves are shown in Figure 9.

## 4. Discussion

The pathogenesis of CHD is complex and is primarily related to lipid metabolism disorders, vascular endothelial injury, platelet aggregation, and thrombosis [34]. Disease progression involves the participation of macrophages, smooth muscle cells, endothelial cells, and other cell types [35]. In recent years, researchers have investigated the prevention and treatment of CHD using TCM [36–38]. YXTMD is an effective prescription for the treatment of CHD, and previous studies have confirmed its therapeutic effects. However, the specific active ingredients and mechanisms of action remain unclear. Network pharmacology can be used to effectively integrate TCM and modern medicine, thereby enabling elucidation of the mechanisms of action of TCM compounds at the molecular level. In the present study, a total of 83 active components of YXTMD and 140 “YXTMD-CHD-BSS” common targets were obtained via network pharmacology. Further analysis showed that YXTMD can act on multiple biological functions associated with CHD with BSS and treat the disease via multiple targets, confirming that YXTMD has the hierarchical network characteristics of being “multi-component, multitarget, and multipathway” in the treatment of CHD with BSS.

The results of our study showed that the core active components of YXTMD in the treatment of CHD with BSS were 5,7,4′-trimethylapigenin, tetramethoxyluteolin, isosinensetin, sinensetin, 5,7-dihydroxy-2-(3-hydroxy-4-methoxyphenyl)chroman-4-one, danshenol B, danshenol A, eriodyctiol, luteolin, naringenin, and kaempferol. The first 10 components belonged to danshen and zhishi. Danshen (Radix Salviae Miltiorrhizae) activates the blood and resolves stasis, and zhishi (Fructus Aurantii Immaturus) regulates qi and dissipates phlegm, consistent with the principle of treating BSS. Most of the active ingredients were flavonoids, which have the effects of antioxidation, anti-inflammation, vasodilation, inhibition of platelet aggregation, and regulation of blood lipid levels, thus exerting beneficial therapeutic effects on cardiovascular and cerebrovascular diseases [39–41]. Modern research has shown that sinensetin can exert various pharmacological effects, including anti-inflammatory and antioxidant effects, by reducing the secretion of inflammatory factors such as IL-1*β*, IL-6, and TNF-*α* [42]. In addition, 5,7-dihydroxy-2-(3-hydroxy-4-methoxyphenyl)chroman-4-one can scavenge oxygen-free radicals and has anti-inflammatory and blood lipid-lowering effects [43]. Danshenol effectively inhibits calcium overload in tissues, thereby reducing myocardial ischemia injury in rats [44]. Luteolin can scavenge reactive oxygen species and reduce oxidative damage in inflammatory cells [45]. It can also regulate inflammatory mediators and inflammatory factors, affecting the cyclooxygenase and lipoxygenase pathways to affect the arachidonic acid pathway, thereby reducing the production of prostaglandins to protect the cardiovascular system and inhibit platelet activity and arterial thrombosis [46]. Naringenin has antioxidant, anti-inflammatory, and antiapoptotic effects [47] and can also inhibit platelet activity and arterial thrombosis [48]. Kaempferol plays an important role in the inflammatory response and can reduce the expression of reduced coenzyme oxidase to inhibit ROS generation, protect protein tyrosine phosphatase-2 (SHP-2), and inhibit platelet activation. It can also prevent CHD as well as other cardiovascular and cerebrovascular diseases [49]. This suggests that YXTMD can treat CHD with BSS by exerting anti-inflammatory, antioxidation, and antithrombotic effects, and regulating lipid metabolism. In this compound, danshen and zhishi are the main drugs that show efficacy and should be considered as important directions for later drug development.

In the present study, we identified 18 key targets of YXTMD for the treatment of CHD with BSS: EGFR, VEGFA, AKT1, STAT3, TP53, ERBB2, PIK3CA, HSP90AA1, MTOR, SRC, CASP3, MMP9, IL2, NRAS, PTPN11, TNF, PTGS2, and FGF2. Previous studies have shown that VEGFA, EGFR, and FGF2 are related to vascular endothelial regeneration, and that vascular endothelial cell damage is a significant feature of atherosclerosis [50]. VEGF can act on vascular endothelial cells and regulate endothelial cell proliferation through the PI3K-Akt signaling pathway, thereby promoting angiogenesis [33]. EGFR is involved in the vascular pathophysiology and oxidative stress of macrophages, and inhibition of EGFR can resist oxidative stress, macrophage infiltration, and proliferation of SMCs in lesions [51]. FGF2 regulates cell differentiation and proliferation and promotes the angiogenic activity of human microvascular endothelial cells [52]. AKT1 is a serine/threonine protein kinase that controls the cell cycle, protein synthesis, and angiogenesis [53]. Akt can regulate various downstream signaling molecules, such as eNOS, which plays an important role in vascular remodeling and relaxation, angiogenesis, and wound healing [32]. Inhibition of the transcription factor STAT3 can mediate increased M2 phenotypic differentiation of macrophages, thereby inhibiting the formation of atherosclerotic plaques [54]. TP53 is a tumor suppressor protein that plays a role in atherosclerosis development as well as the growth and death of vascular smooth muscle cells by regulating cellular senescence, proliferation, and apoptosis [55]. ERBB2 is a tyrosine kinase receptor, and a previous study showed that activation of the NRG–ERBB pathway can promote the regeneration of cardiomyocytes, thereby repairing damaged myocardial function [56]. The mTOR protein is a serine/threonine protein kinase downstream of PI3K-Akt that is involved in regulating cell survival, apoptosis, and proliferation [57]. SRC is involved in various biological processes including cell proliferation, movement, and migration. It can activate the phosphorylation of the Y357 site on yes-related proteins, thereby regulating the Gp130 protein to promote cardiomyocyte proliferation during cardiac regeneration [58]. CASP3 is the initiator and executor of apoptosis. A previous study has shown that CASP3 can regulate oxidative stress damage to a certain extent, thereby reducing myocardial damage [59]. Moreover, TNF, IL2, MMP9, and PTGS2 play important roles in the inflammatory response. TNF is a tumor necrosis factor that can also promote atherosclerosis by increasing the endocytosis of LDL in endothelial cells, thereby promoting the deposition of LDL in the vascular walls [60]. IL2 is an inflammatory factor that is related to the formation of atherosclerosis. MMP9 is a matrix metalloproteinase that is involved in various pathological processes, such as inflammation and atherosclerosis. PTGS2 converts arachidonic acid to prostaglandins and is overexpressed under mechanical, chemical, and physical stimulation, thereby promoting the development of an inflammatory response. The molecular docking results of this study also showed that the core active components of YXTMD could bind well to the key targets AKT1 and VEGFA, which can be used as important indicators for future research.

In the present study, GO functional and KEGG enrichment analyses revealed that YXTMD primarily targets the PI3K-Akt signaling pathway, proteoglycan in cancer, Rap1 signaling pathway, MAPK signaling pathway, microRNAs in cancer, and lipids and atherosclerosis in the treatment of CHD with BSS. The primary biological processes involved included wound healing, regulation of body fluid levels, and vascular progress in the circulatory system. The PI3K-AKt pathway plays an important role in growth in vivo, and can activate antiapoptotic mechanisms, glucose metabolism, protein synthesis, and other processes to promote cell proliferation [61]. It also plays an important role in the regulation of cardiomyocytes, survival, and function [62]. The PI3K-AKt pathway can also regulate the inflammatory response and oxidative stress injury, which are closely related to the formation of atherosclerosis [63]. AKT1 is the center of the PI3K-AKt signaling pathway, and inhibition of its overactivation can alleviate high-fatdiet-induced atherosclerosis in ApoE + mice [64]. It participates in various biological processes, such as cell metabolism, proliferation, and survival, by regulating various downstream signaling molecules [65]. The downstream targets of the PI3K-AKt pathway include eNOS, NF-*κ*B, and GSK-3*β*. Activated Akt can phosphorylate eNOS, thereby promoting the production of endogenous NO, accelerating the regeneration of vascular endothelial cells, and dilating blood vessels. NF-*κ*B promotes cell proliferation, inhibits apoptosis, and is an important inflammatory activator [66]. GSK-3*β* is a multifunctional serine/threonine protein kinase that negatively regulates itself by activating the PI3K-Akt pathway, thereby mediating cell metabolism, proliferation, differentiation, apoptosis, and other biological processes [67]. Accordingly, regulation of these target molecules can promote the regeneration of vascular endothelial cells, reduce inflammation, resist oxidative stress, and regulate carbohydrate and lipid metabolism. Based on these results, we speculated that the PI3K-AKt pathway was closely related to the treatment of CHD with BSS by YXTMD.

Based on previous research from our group and the pathogenesis of CHD with BSS, we further verified the accuracy of the network pharmacology results and more intuitively reflected the clinical efficacy and specific molecular mechanism of YXTMD in the treatment of CHD with BSS through a clinical trial. In the trial, we determined the effects of the clinical efficacy, blood lipid level, endothelial injury marker index (NO), inflammatory factor index (IL-1*β* and TNF-*α*), oxidative stress indicators (MDA and SOD), and the PI3K-AKt pathway and its downstream proteins (PI3k, AKt, NF-*κ*B, eNOS, and GSK-3*β*) in patients with CHD with BSS. Results showed that after treatment, the clinical curative effect of the treatment group was better than that of the control group. YXTMD improved the curative effect scores of patients with BSS and reduced the serum TC and LDL-C levels. PCR results showed that, compared with the control group, the serum levels of PI3k and AKt mRNA significantly increased, and the levels of GSK-3*β* mRNA significantly decreased in the treatment group; however, the levels of *NF-κB* and *eNOS* mRNA did not significantly change. ELISA results showed no significant changes in serum MDA, SOD, NO, and TNF-*α* levels in the two groups before and after treatment, and the serum IL-1*β* level in the control group was higher than before treatment. The above results demonstrate that YXTMD was clinically effective in treating CHD with BSS. It can improve the efficacy score of BSS and reduce blood lipid levels. The specific mechanism may be related to the activation of the PI3K/Akt signaling pathway, downregulation of GSK-3*β*, and regulation of lipid metabolism.

Notably, this study has some limitations. Preliminary research results showed that the main active components of YXTMD have anti-inflammatory, antioxidant, vasodilatory, antithrombotic, and lipid-metabolism-regulating effects. However, the results of later clinical trials have revealed that YXTMD activates the PI3K/Akt signaling pathway and is primarily involved in regulating lipid metabolism. Its anti-inflammatory, antioxidant, and vasodilatory effects were not obvious, which may be explained by the following factors: (1) This trial was based on a heterogeneous human population, which involves many uncontrollable factors. (2) The difficulty in collecting clinical samples and the problem of patient compliance resulted in a small sample size. (3) The subjects of this study were all patients with BSS. Modern studies have shown that increased blood lipids and viscosity are the biochemical basis for phlegm and blood stasis. This occurs when a large amount of lipids condense in the veins to form phlegm turbidity, and the phlegm is stuck in the veins for a prolonged period and condenses into blocks, leading to endogenous blood stasis. Therefore, BSS formation was closely related to blood lipid levels. These factors affected the trial results to some extent, so large-scale clinical studies or in-depth studies at the animal and cellular levels are needed at a later stage to explore the specific mechanism by which YXTMD treats CHD with BSS.

## 5. Conclusions

Our study explored the mechanism of action of YXTMD in the treatment of CHD with BBS through a combination of network pharmacology and molecular docking. The results demonstrated that 5,7,4′-trimethoxyflavone, tetramethoxyluteolin, isosinensetin, sinensetin, and 5,7-dihydroxy-2-(3-hydroxy-4-methoxyphenyl)chroman-4-one may be the main active components of YXTMD. These components act on key targets, such as EGFR, VEGFA, AKT1, STAT3, TP53, ERBB2, and PIK3CA, in the treatment of CHD with BBS. YXTMD had the characteristics of being multicomponent, multitarget, and multipathway in treating CHD with BBS. Clinical trial results showed that the mechanism of action of YXTMD in treating CHD with BBS may be related to the activation of the PI3K-AKt signaling pathway, downregulation of GSK-3*β*, and mediation of lipid-metabolism-based metabolic processes. These results provide a theoretical basis for the clinical application of YXTMD and highlight directions for follow-up studies on the development of anti-CHD drugs.

## Figures and Tables

**Figure 1:** The workflow used in the study.

**Figure 2:** Venn diagram showing the common targets of “YXTMD-CHD-BSS.”

**Figure 3:** “YXTMD active components-common targets” network. Note. The red dots represent danshen, pink dots represent zhishi, yellow dots represent guizhi, purple dots represent renshen, and green dots represent zexie. Blue dots represent the common target.

**Figure 4:** Diagrams of the PPI network and subnetwork topology analysis of common targets. (a) Protein–protein interaction network. (b) Subnetwork topology analysis diagram. Yellow nodes are the core genes obtained after screening.

**Figure 5:** GO functional analysis.

**Figure 6:** KEGG enrichment analysis.

**Figure 7:** Visualization of the PI3K-Akt signaling pathway.

**Figure 8:** Results of molecular docking. Structures show molecular docking of (a) AKT1-5,7,4′-trimethylapigenin, (b) AKT1-tetramethoxyluteolin, (c). AKT1-5,7-dihydroxy-2-(3-hydroxy-4-methoxyphenyl)chroman-4-one, (d) VEGFA-5,7,4′-trimethylapigenin, (e) VEGFA-tetramethoxyluteolin, and (f) VEGFA-5,7-dihydroxy-2-(3-hydroxy-4-methoxyphenyl)chroman-4-one.

**Figure 9:** Amplification plots and melting curves.

**Table 1:** Primer sequences.

Gene	Sequences (5′⟶3′)	Length (bp)
GAPDH	Forward ACAGCCTCAAGATCATCAGC	104
	Reverse GGTCATGAGTCCTTCCACGAT	

eNOS	Forward ACCCTCACCGCTACAACATCC	102
	Reverse TGATTTCCACTGCTGCCTTGTCT	

AKT1	Forward AGCCCTGGACTACCTGCACTCG	98
	Reverse CTGTGATCTTAATGTGCCCGTCCT	

PI3K	Forward TGCGTCTACTAAAATGCATGG	122
	Reverse AACTGAAGGTTAATGGGTCA	

GSK-3*β*	Forward GCACATCCTTGGACTAAGGTC	229
	Reverse CCAGAGGTGGATTACTTGACAG	

NF-*к*B-p65	Forward CGCCTGTCCTTTCTCATCCCAT	141
	Reverse CCTCTTTCTGCACCTTGTCACAC	

**Table 2:** Node degree ranking of main active compounds.

Compound Id	Compound name	Degree	Source
MOL013279	5,7,4′-trimethylapigenin	32	*Fructus Aurantii Immaturus*
MOL007879	Tetramethoxyluteolin	31	*Fructus Aurantii Immaturus*
MOL013277	Isosinensetin	30	*Fructus Aurantii Immaturus*
MOL001803	Sinensetin	29	*Fructus Aurantii Immaturus*
MOL005100	5,7-dihydroxy-2-(3-hydroxy-4-methoxyphenyl)chroman-4-one	28	*Fructus Aurantii Immaturus*
MOL007081	Danshenol B	27	Radix *Salviae Miltiorrhizae*
MOL007082	Danshenol A	27	Radix *Salviae Miltiorrhizae*
MOL002914	Eriodyctiol (flavanone)	27	*Fructus Aurantii Immaturus*
MOL000006	Luteolin	26	Radix *Salviae Miltiorrhizae* and *Fructus Aurantii Immaturus*
MOL004328	Naringenin	26	*Fructus Aurantii Immaturus*
MOL000422	Kaempferol	26	Radix Ginseng

**Table 3:** Integration of key genes using Degree and CytoNCA algorithms.

Name	Betweenness	Closeness	Degree	Eigenvector	LAC	Network
EGFR	12.49	1.00	34	0.31	21.88	32.46
VEGFA	10.56	0.94	32	0.29	20.75	28.75
AKT1	11.55	0.94	32	0.29	20.25	28.34
STAT3	10.56	0.94	32	0.29	20.75	28.75
TP53	6.63	0.85	28	0.26	19.43	23.71
ERBB2	6.58	0.81	26	0.24	16.92	19.96
PIK3CA	2.16	0.77	24	0.24	18.67	20.35
HSP90AA1	2.56	0.77	24	0.24	18.33	19.81
MTOR	1.80	0.74	22	0.22	17.09	17.90
SRC	2.14	0.74	22	0.22	16.73	17.66
CASP3	2.55	0.74	22	0.21	16.73	18.00
MMP9	2.71	0.74	22	0.21	16.36	17.93
IL2	3.46	0.74	22	0.21	15.64	16.60
NRAS	3.54	0.74	22	0.21	14.91	15.94
PTPN11	1.84	0.71	20	0.20	14.80	15.73
TNF	2.02	0.71	20	0.19	15.20	16.30
PTGS2	0.69	0.68	18	0.18	14.67	15.53
FGF2	2.16	0.68	18	0.18	12.44	13.18

**Table 4:** Molecular docking (unit: kcal/mol).

Number	Molecule name	Molecular formula	AKT1	VEGFA
1	5,7,4′-trimethylapigenin	C18H16O5	−8.5	−6.8
2	Tetramethoxyluteolin	C19H18O6	−8.8	−6.7
3	Isosinensetin	C20H20O7	−8.2	−6.8
4	Sinensetin	C20H20O7	−8.1	−6.3
5	5,7-dihydroxy-2-(3-hydroxy-4-methoxyphenyl)chroman-4-one	C16H14O6	−8.5	−7.1

**Table 5:** Comparison of ECG effective rate between the two groups (%).

Groups	*N*	Markedly effective	Effective	Ineffective	Total effective rate (%)
Treatment group	4	2 (50)	2 (50)	0 (0)	100
Control group	6	1 (16.7)	2 (33.3)	3 (50)	50

**Table 6:** Comparison of blood stasis syndrome scores between the two groups ($\bar{x}$ ± *s*).

Groups	*N*	Before treatment	After treatment	*P* value
Treatment group	7	35.71 ± 9.09	19.29 ± 7.30	<0.05^*∗*^
Control group	7	31.71 ± 8.83	27.43 ± 10.08	0.182
*P* Value		0.396	<0.05^#^	

*Note*. ^*∗*^*P* < 0.05 compared to pretreatment; ^#^*P* < 0.05 compared to the control group after treatment.

**Table 7:** Comparison of blood lipids before and after treatment between the two groups ($\bar{x}$ ± *s*, *n* = 7).

Items	Treatment group		Control group	
	Before treatment	After treatment	Before treatment	After treatment
TC	3.63 ± 1.07	3.41 ± 0.81^#^	3.82 ± 0.69	4.38 ± 0.51^*∗*^
TG	1.41 ± 0.68	1.33 ± 0.60	2.24 ± 1.28	1.88 ± 0.83
LDL-C	2.50 ± 0.97	2.14 ± 0.78^#^	2.54 ± 0.54	2.99 ± 0.48^*∗*^
HDL-C	0.97 ± 0.29	1.11 ± 0.27^*∗*^	0.99 ± 0.27	1.21 ± 0.33^*∗*^

Note. ^*∗*^*P* < 0.05 compared to pretreatment; ^#^*P* < 0.05 compared to the control group after treatment.

**Table 8:** Comparison of serum levels of MDA, SOD, NO, TNF-*α*, and IL-1*β* before and after treatment between the two groups ($\bar{x}$ ± *s*, *n* = 7).

Items	Treatment group		Control group	
	Before treatment	After treatment	Before treatment	After treatment
MDA	0.11 ± 0.01	0.11 ± 0.01	0.12 ± 0.01	0.13 ± 0.01
SOD	0.20 ± 0.06	0.25 ± 0.05	0.19 ± 0.03	0.22 ± 0.02
NO	4.89 ± 1.91	6.10 ± 2.57	6.13 ± 2.81	7.93 ± 2.53
IL-1*β*	15.76 ± 3.92	12.57 ± 4.04	15.50 ± 2.79	18.60 ± 2.86^*∗*^
TNF-*α*	16.66 ± 2.19	16.30 ± 0.99	18.57 ± 3.17	19.30 ± 2.91

Note. ^*∗*^*P* < 0.05 Compared to pretreatment.

**Table 9:** Comparison of the levels of *PI3k*, *AKt*, *NF-KB*, *eNOS*, and *GSK-3β* mRNA before and after treatment between the two groups ($\bar{x}$ ± *s*, *n* = 7).

Items	Treatment group		Control group	
	Before treatment	After treatment	Before treatment	After treatment
PI3k	1.43 ± 0.85	3.03 ± 0.38^*∗*^^#^	1.04 ± 0.49	1.70 ± 0.72^*∗*^
Akt	1.05 ± 0.33	3.43 ± 1.04^*∗*^^#^	1.16 ± 0.77	2.20 ± 0.81^*∗*^
NF-*κ*B	0.90 ± 0.42	2.51 ± 0.85^*∗*^	0.99 ± 0.43	1.85 ± 0.73^*∗*^
eNOS	0.80 ± 0.21	1.76 ± 0.58^*∗*^	0.86 ± 0.29	1.32 ± 0.41^*∗*^
GSK-3*β*	1.34 ± 0.35	0.35 ± 0.94^*∗*^^#^	1.07 ± 0.39	0.80 ± 0.29

Note. ^*∗*^*P* < 0.05 compared to pretreatment; ^#^*P* < 0.05 compared to the control group after treatment.

## Data Availability

All data obtained or analyzed during this study are included within the article.
